The article "CMMCSegNet: Cross-Modality Multicascade Indirect LGE Segmentation on Multimodal Cardiac MR" was published in 2021. Journal: Comput Math Methods Med.

# CMMCSegNet: Cross-Modality Multicascade Indirect LGE Segmentation on Multimodal Cardiac MR

**DOI:** 10.1155/2021/9942149

**Published:** 2021-06-05

**Authors:** Yu Wang, Jianping Zhang

**Affiliations:** School of Mathematics and Computational Science, Xiangtan University, Xiangtan, Hunan 411105, China

## Abstract

Since Late-Gadolinium Enhancement (LGE) of cardiac magnetic resonance (CMR) visualizes myocardial infarction, and the balanced-Steady State Free Precession (bSSFP) cine sequence can capture cardiac motions and present clear boundaries; multimodal CMR segmentation has played an important role in the assessment of myocardial viability and clinical diagnosis, while automatic and accurate CMR segmentation still remains challenging due to a very small amount of labeled LGE data and the relatively low contrasts of LGE. The main purpose of our work is to learn the real/fake bSSFP modality with ground truths to indirectly segment the LGE modality of cardiac MR by using a proposed cross-modality multicascade framework: cross-modality translation network and automatic segmentation network, respectively. In the segmentation stage, a novel multicascade pix2pix network is designed to segment the fake bSSFP sequence obtained from a cross-modality translation network. Moreover, we propose perceptual loss measuring features between ground truth and prediction, which are extracted from the pretrained vgg network in the segmentation stage. We evaluate the performance of the proposed method on the multimodal CMR dataset and verify its superiority over other state-of-the-art approaches under different network structures and different types of adversarial losses in terms of dice accuracy in testing. Therefore, the proposed network is promising for Indirect Cardiac LGE Segmentation in clinical applications.

## 1. Introduction

Multimodal CMR imaging is an essential tool in clinics for the screening and diagnosis of cardiac diseases. Different imaging modalities contain different sorts of useful information for cardiac disease screening task; the combination of different imaging modalities can overcome the limitations of an individual modality. The contrast agent for the LGE MR imaging is injected for 10-20 minutes; LGE images with distinctive locally brightness compared with the healthy tissues can enhance myocardial necrosis or scarring, which is a standard practice to evaluate cardiac structure, cardiac function, myocardial perfusion, and myocardial activity. Different from LGE images, the bSSFP can highlight the high signal area of the fluid but appear a uniform signal for other tissues; e.g., the large blood vessels and coronary arteries can be observed clearly in bSSFP because of more obvious contrast in the heart muscle and blood pool. T2-weighted MRI is effective in reducing false-positive results. Considering different MRI modalities is thus important for the acquisition of accurate cardiac information [1].

Segmentation of multimodal CMR images is a critical step in the process for the following diagnosis and surgical planning. However, it takes 20 minutes/case for an experienced doctor to manually segment the LGE images, it is extremely time-consuming to manually identify and delineate the corresponding structure in cardiac, and the result depends on the professional ability of doctors and varies from person to person. Therefore, the development of automatic and reliable LGE image segmentation algorithms is of high clinical values for patients suffering from myocardial infarction.

Tao and Der Geest proposed a method for segmenting the LGE images using myocardial morphological information [2]. Popescu et al. used a mask SLIC clustering method and Otsu threshold to segment LGE images [3]. In recent years, deep learning has achieved remarkable success in computer vision. More and more image processing methods are based on the CNN model [4, 5]. Chen et al. [6] proposed to use the domain adaption to fuse the features of unlabeled LGE images and then use the fused features to train the segmentation network. In addition, many approaches based on attention mechanisms [7, 8] and multiview methods [9] have been developed recently for segmenting medical images. Yang et al. combined multiview and attention mechanism to segment cardiac LGE images [10]. An automatic cardiac LGE segmentation algorithm based on the CNN is far more efficient and robust, and commonly more accurate than traditional methods [11, 12], so it is necessary to automatically segment the LGE images.

However, automatic LGE CMR segmentation is still arduous. Besides the great variations of the location and geometry of the heart region across different patients, Zhuang [1] pointed three major challenges related to the intensity distributions of the LGE CMR modality: (i) the intensity range of myocardium in LGE imaging leads to indistinguishable boundaries from its adjacent organs; (ii) the pathologies result in heterogeneous intensity of the myocardium, making the assumption of a simple distribution such as the single component Gaussian density invalid; and (iii) the preprocessing enhancement for the LGE CMR modality can be complex. So it is more difficult to segment directly LGE modality, especially in case of a small amount of labeled LGE data.

GAN was first proposed by Goodfellow et al. [13] for image synthesis, which uses a generator network and discriminator network, to pit one against the other (thus the “adversarial”) in order to generate fake synthetic instance that can pass for real data. Here, the generator generates a fake image by random noise, the discriminator judges whether the input data is true (data comes from real labels) or false (the data comes from the output of the generator). The aim of GANs is to learn the underlying distribution of training data in order to generate data that the discriminator cannot distinguish. At the same time, the game between the generator and the discriminator reaches the Nash equilibrium, i.e., the generated data distribution *p*_*g*_ is equal to real data distribution *p*_*d*_. With the development of GANs [14], such models are widely used in image processing, including image and video generation [15], image segmentation [16], image synthesis [17], and image super resolution [18].

In this work, we propose a novel cross-modality multicascade framework for indirect LGE segmentation (CMMCSegNet), which is trained on multimodal cardiac MR data with a very small amount of LGE labels (for the LGE modality in Multisequence Cardiac MR Segmentation Challenge 2019 datasets [1], only five patients are labeled). The main contributions of this work are clarified as follows:

1. We develop a novel indirect LGE segmentation framework based on multimodal images; one of the primary components is to translate the LGE modality that needs to be segmented but only has very small amount of labeled data, into the bSSFP modality that is easy to be segmented by our proposed method
2. We propose a multicascade pix2pix network for image segmentation; that is, the generator is formed by cascading multiple subnetworks. In the segmentation network, we regard segmentation as the translation process from the original image to the segmentation target
3. We employ the perceptual loss that uses a pretrained VGG19 network to compare the feature differences between the labels and generation during the proposed multicascade pix2pix network training

The rest of this work is organized as follows. We first give some preliminaries in Section 2. We describe our CMMCSegNet in details in Section 3. We give experimental results in Section 4. Finally, we conclude this work in Section 5.

## 2. Related Works

Tissue or organ segmentation plays an important role in the field of medical image processing. Medical image segmentation has been explored extensively; however, challenges in generality, robustness, and efficiency still remain. For brevity, we only focus below on the most closely related works.

### 2.1. Cascade Structure

A cascading network is to connect multiple subnetworks together to form a multilevel network. The cascading method has been effectively used in many vision applications like classification [19], image translation [20], detection [21], super resolution [22], and semantic segmentation [23]. For example, Cui et al. proposed a deep cascade network for image super resolution [22]. Cai and Vasconcelos proposed the use of cascade structure for object detection [21]. Zhao et al. proposed the recursive cascaded networks for medical image registration [24]. Armanious et al. proposed the use of cascaded generator network for image translation [20]. Havaei et al. proposed a new cascade architecture for brain tumor segmentation [23]. Li et al. [25] proposed to classify easy regions in a shallow network and train deeper networks to deal with hard regions. Lin et al. [26] proposed a top-down architecture with lateral connections to propagate deep semantic features to shallow layers.

Different from previous cascade networks, the multicascade pix2pix network proposed in this paper is a multiple U-net cascade structure for image segmentation, which allows an innovative way to supervise each generator individually for pix2pix GANs. To our best knowledge, this is an early and original attempt to adopt a cascade architecture in pix2pix GAN-based medical image segmentation. We will introduce more details in Section 3.

### 2.2. Multimodal Cardiac MR Image Segmentation

Recent literature suggests two main approaches to complete multimodal CMR image segmentation. One popular approach is about the GAN strategy based on cross-modality image translation that refers to the translation of images with modality *𝒳* into images with modality *𝒴*, which plays an increasingly important role in computer vision. Isola et al. [18] proposed the use of conditional GAN to implement a paired image-to-image translation. Ben-Cohen et al. used CT images to synthesize PET images based on the pix2pix network [27]. Cycle-GAN [28] was proposed for unpaired image-to-image translation. BiCycle-GAN [29] solved the translation process from single image to multicategory image. In addition, some GAN networks including DualGAN [30] and UNIT [31] were also proposed for unpaired image-to-image translation.

In CMR datasets [1], MR images of the different modalities are not strictly matched, so the classical unpaired image-to-image translation [32] can be applied to cross-modality CMR segmentation. Chen et al. [33] proposed to use UNIT to translate bSSFP images into LGE images and then train the segmentation network where the LGE images are provided by the translation architecture. Campello et al. also proposed to use Cycle-GAN to translate bSSFP images into LGE images but train the U-net network [34] for LGE segmentation. Tao et al. [35] proposed to integrate the translation network (Cycle-GAN) with the segmentation network to achieve LGE image segmentation.

Another promising approach is about the strategy on image registration. Roth et al. proposed to register LGE images with ground truths into LGE images without ground truths, after multiatlas label fusion by majority voting; they obtained a noisy LGE label and then trained a LGE segmentation network [36]. Liu et al. proposed a registration method for histogram matching to achieve augmentation of the LGE images [37].

## 3. Proposed Cross-Modality SegNet

The goal of this work is to achieve cardiac segmentation for LGE modality where a small amount of samples are labeled. Our CMMCSegNet (https://github.com/wangyu719/CmmcSegNet) framework is designed to facilitate indirect segmentation for the multimodal CMR images. The total framework is shown in Figure 1, including a training architecture and a testing architecture.

Our datasets are from Multisequence Cardiac MR Segmentation Challenge 2019 datasets (MS-CMRSeg 2019) [1]. In this work, we use LGE modality with 45 patients and bSSFP modality with 35 annotated patients (see Figure 2 for more details). Only five ground truth annotations are available in LGE modality of MS-CMRSeg 2019 datasets; hence, it is difficult to directly segment LGE modality using deep CNN-based methods. Figure 2 shows the differences between LGE and bSSFP images from the same patient. Furthermore, it is found that the bSSFP modality has a more obvious contrast than LGE modality, so we believe that the bSSFP is easier to be segmented. Besides, the bSSFP modality has a large number of images (35 patients) with ground truth annotations, so it is not difficult to train the bSSFP modality using the deep learning-based method.

### 3.1. Cross-Modality Image Translation

One of the primary components in training architecture is a cross-modality translation network, which can be trained end-to-end with unpaired modalities. Before segmenting the bSSFP images to achieve indirect segmentation of LGE images, we first present a Cycle-GAN architecture of translating LGE into bSSFP images.

Inspired by the knowledge distillation between unpaired image-to-image translation networks [32], we employ Cycle-GAN to achieve cross-modality image translation for CMR datasets. Let *𝒳*, *𝒴* be two image domains that represent the LGE and bSSFP modalities, respectively. *G*_*A*_^*t*^ : *𝒳*⟶*𝒴* and *G*_*B*_^*t*^ : *𝒴*⟶*𝒳* are two generators of the cross-modality translation network such that *G*_*A*_^*t*^ and *G*_*B*_^*t*^ are inverse mappings of each other; that is, *G*_*B*_^*t*^(*G*_*A*_^*t*^(*I*_*𝒳*_)) ≈ *I*_*𝒳*_, *G*_*A*_^*t*^(*G*_*B*_^*t*^(*I*_*𝒴*_)) ≈ *I*_*𝒴*_ for any unpaired images *I*_*𝒳*_ ∈ *𝒳*, *I*_*𝒴*_ ∈ *𝒴*. *D*_*A*_^*t*^ and *D*_*B*_^*t*^ are the discriminators of the cross-modality translation network, to distinguish that the input of discriminator is real or fake.

The Cycle-GAN architecture implementing cross-modality image translation for unpaired LGE/bSSFP datasets consists of two cycles: LGE cycle and bSSFP cycle. In the LGE cycle, the first generator (*G*_*A*_^*t*^) is trained to transform LGE modality into fake bSSFP modality, the second generator (*G*_*B*_^*t*^) is trained to transform the generated fake bSSFP modality back to the original LGE modality, and the discriminator *D*_*A*_^*t*^ discriminates between real and synthesized bSSFP modalities. In fact, enlightened by the activation-based attention transfer strategies, the discriminator *D*_*A*_^*t*^ is designed to extract the supervision information that modulates the learning of the generator *G*_*A*_^*t*^. In the bSSFP cycle, real bSSFP was transformed to fake LGE by using the generator *G*_*B*_^*t*^, the generator *G*_*A*_^*t*^ transforms the generated LGE to the original bSSFP, and the discriminator *D*_*B*_^*t*^ discriminates between real and fake bSSFP modality. Finally, the network framework is shown in Figure 1(b).

The overall training loss of our translation network is defined as

(1) $$\begin{array}{c} \left(G_{A}^{t*},G_{B}^{t*};D_{A}^{t*},D_{B}^{t*}\right)=\arg\;\min\;\max_{\left(G_{A}^{t},G_{B}^{t}\right),\left(D_{A}^{t},D_{B}^{t}\right)}\left\{L^{t}\left(G_{A}^{t},G_{B}^{t};D_{A}^{t},D_{B}^{t}\right)≕\lambda_{1}L_{\text{cyc}}\left(G_{A}^{t},G_{B}^{t}\right)+L_{\text{gan}}\left(G_{A}^{t},D_{A}^{t},X,Y\right)+L_{\text{gan}}\left(G_{B}^{t},D_{B}^{t},X,Y\right)\right\}, \end{array}$$

where *ℒ*_gan_(*G*_*A*_^*t*^, *D*_*A*_^*t*^, *𝒳*, *𝒴*) and *ℒ*_gan_(*G*_*B*_^*t*^, *D*_*B*_^*t*^, *𝒳*, *𝒴*) are two adversarial losses defined by

(2) $$\begin{array}{c} L_{\text{gan}}\left(G_{A}^{t},D_{A}^{t},X,Y\right)=E_{I_{Y}\sim p_{d\left(I_{Y}\right)}}\left[\log\left(D_{A}^{t}\left(I_{Y}\right)\right)\right]+E_{I_{X}\sim p_{d\left(I_{X}\right)}}\left[\log\left(1-D_{A}^{t}\left(G_{A}^{t}\left(I_{X}\right)\right)\right)\right],\\ L_{\text{gan}}\left(G_{B}^{t},D_{B}^{t},X,Y\right)=E_{I_{X}\sim p_{d\left(I_{X}\right)}}\left[\log\left(D_{B}^{t}\left(I_{X}\right)\right)\right]+E_{I_{Y}\sim p_{d\left(I_{Y}\right)}}\left[\log\left(1-D_{B}^{t}\left(G_{B}^{t}\left(I_{Y}\right)\right)\right)\right], \end{array}$$

and the generation similarity *ℒ*_cyc_(*G*_*A*_^*t*^, *G*_*B*_^*t*^) is defined by

(3) $$\begin{array}{c} L_{\text{cyc}}\left(G_{A}^{t},G_{B}^{t}\right)=E_{I_{X}\sim p_{d\left(I_{X}\right)}}\left[{\left\|G_{B}^{t}\left(G_{A}^{t}\left(I_{X}\right)\right)-I_{X}\right\|}_{1}\right]+E_{I_{Y}\sim p_{d\left(I_{Y}\right)}}\left[{\left\|G_{A}^{t}\left(G_{B}^{t}\left(I_{Y}\right)\right)-I_{Y}\right\|}_{1}\right], \end{array}$$

and *λ*_1_ is the weight parameter for balancing the contributions of the generation loss *ℒ*_cyc_(*G*_*A*_^*t*^, *G*_*B*_^*t*^) and the two adversarial losses *ℒ*_gan_(*G*_*A*_^*t*^, *D*_*A*_^*t*^, *𝒳*, *𝒴*) and *ℒ*_gan_(*G*_*B*_^*t*^, *D*_*B*_^*t*^, *𝒳*, *𝒴*).

### 3.2. Multicascade pix2pix Segmentation

Recently, the GAN-based framework is proposed to segment the retinal vessel [38]. We understand image segmentation as the translation from paired image to image (from an original image to a predicted segmentation results); hence, we propose a new image segmentation method using a multicascade technique and pix2pix structure, which we call a multicascade pix2pix network.

#### 3.2.1. Multicascade Network

Our multicascade pix2pix segmentation network shown in Figure 1(c) is based on the GAN architecture, which consists of multiple generators *G*_*k*_^*s*^ (*k* = 1, ⋯, *n*) and a shared discriminator *D*^*s*^.

The generator *G*_1_^*s*^: *𝒴*⟶*𝒮* translates *I*_*𝒴*_ to *I*_*𝒮*_^1^, where the original input *I*_*𝒴*_ ∈ *𝒴* is 1 × 256 × 256 real or fake bSSFP image, and the first generation *I*_*𝒮*_^1^ ∈ *𝒮* is a prediction for the corresponding label. The other generators *G*_*k*_^*s*^: *𝒮*⟶*𝒮*(*k* = 2, ⋯, *n*) furtherly improve the previous predicted probability *I*_*𝒮*_^*k*−1^ to obtain more optimal prediction

(4) $$\begin{array}{c} I_{S}^{k}≔G_{k}^{s}\circ G_{k-1}^{s}\circ \cdots \circ G_{1}^{s}\left(I_{Y}\right), \end{array}$$

where *I*_*𝒴*_ and *I*_*𝒮*_^*k*^ have the same size. In this work, *G*_*k*_^*s*^ is formed by the U-net [5] or ResNet [39] network for the purpose of more accurate segmentation. In experimental evaluation, we will compare the effects of different generator networks on the segmentation results. The purpose of this network is to obtain the final segmented result *I*_*𝒮*_^*f*^ of the original input *I*_*𝒴*_, which also is the result of the LGE segmentation. Therefore, the generated prediction obtained from the multicascade pix2pix segmentation network can be denoted as

(5) $$\begin{array}{c} I_{S}^{f}≔I_{S}^{n}=G_{n}^{s}\circ G_{n-1}^{s}\circ \cdots \circ G_{1}^{s}\left(I_{Y}\right). \end{array}$$

The discriminator *D*^*s*^ is a binary classifier based on pixels or patch-images which provides a network learning-based stopping criterion during generating. For the discriminator *D*^*s*^ in our multicascade pix2pix segmentation network, we employ a convolutional Patch-GAN [18] to distinguish real or fake between the prediction *I*_*𝒮*_^*k*^ and the ground truth *I*_*ℒ*_, where *I*_*𝒮*_^*k*^ is divided into *ℓ* × *ℓ* patches with overlapping images, and each patch is discriminated with those of the ground truth *I*_*ℒ*_, respectively; finally, a 2D probability map is obtained as the discriminator outputs.

To train an optimal segmentation network, the measures between *I*_*𝒮*_^*k*^ and target label *I*_*ℒ*_ can be estimated and minimized to update discriminator *D*^*s*^ that enforces to discriminate the generation and the ground truth. The segmentation network we propose is a conditional version of pix2pix GAN with the multicascade architecture, so the adversarial input in *D*^*s*^ is mainly composed of there components, where the first component is the source image *I*_*𝒴*_ used as the condition and the others are the generation *I*_*𝒮*_^*k*^ and the ground truth *I*_*ℒ*_. At the same time, each generator *G*_*k*_^*s*^ is also optimized to generate domain-invariant representations *I*_*𝒮*_^*k*^ that confuses the discriminator *D*^*s*^.

#### 3.2.2. Loss Functions in Segmentation Stage

The dice score and Jaccard index are commonly used as metrics for the evaluation of image segmentation task. CNNs trained for image segmentation task are usually optimized by minimizing a weighted cross-entropy. In this work, we employ a specially designed loss function *ℒ*^*s*^ to simultaneously measure the generation similarity and the adversarial error, which contains three types of loss functions: adversarial loss *ℒ*_gan_, *ℒ*_1_ loss, and perceptual loss *ℒ*_vgg_.

The original adversarial loss (Vanilla GAN loss) is given by the Kullback-Leibler (KL) divergence score as

(6) $$\begin{array}{c} L_{\text{gan}}\left(\left\{G_{1}^{s},\cdots ,G_{n}^{s}\right\},D^{s}\right)=\overset{n}{\underset{k=1}{\sum }}\omega_{k}^{L_{g}}\left(E_{I_{Y},I_{L}\sim p_{d\left(I_{Y},I_{L}\right)}}\left[\log\left(D^{s}\left(I_{Y},I_{L}\right)\right)\right]+E_{I_{Y}\sim p_{d\left(I_{Y}\right)}}\left[\log\left(1-D^{s}\left(I_{Y},I_{S}^{k}\right)\right)\right]\right), \end{array}$$

where *ω*_*k*_^*ℒ*_*g*_^(*k* = 1, ⋯, *n*) is the given weight enforcing the trade-off between the *n* cascade cross-entropy losses and *I*_*𝒴*_ is a condition input of each convolutional Patch-GAN in our multicascade pix2pix segmentation network. Recently, the most commonly used adversarial losses are WGAN-GP [40] and LSGAN [41]. In the next section, we will compare the performances of three different adversarial losses in our experiments.

*ℒ*_1_ loss is a weighted sum of the absolute distance between the calculated output data *I*_*𝒮*_^*k*^ in the *k*-th cascade block and the ground truth *I*_*ℒ*_, which can make the segmentation results closer to the real results [18], and is defined by

(7) $$\begin{array}{c} L_{1}\left(G_{1}^{s},\cdots ,G_{n}^{s}\right)=\overset{n}{\underset{k=1}{\sum }}\omega_{k}^{L_{1}}\left(E_{I_{Y}\sim p_{d\left(I_{Y}\right)}}\left[{\left\|I_{L}-I_{S}^{k}\right\|}_{1}\right]\right), \end{array}$$

where *ω*_*k*_^*ℒ*_1_^(*k* = 1, ⋯, *n*) are weight constants. Without loss of generality, we will take *ω*_*k*_^*ℒ*_*g*_^ = *ω*_*k*_^*ℒ*_1_^ for all *k* = 1, ⋯, *n* in our experiments.

Besides, we also employ the perceptual loss in our multicascade pix2pix segmentation network, which is composed of a pretrained VGG19 network and is first proposed in image super resolution application [42]. The perceptual loss focuses on feature maps between the output data and the ground truth [43]. It can hence be computed by

(8) $$\begin{array}{c} L_{\text{vgg}}\left(I_{L},\left\{G_{1}^{s},\cdots ,G_{n}^{s}\right\}\right)=\overset{n,M,N_{i}}{\underset{k,i,j=1}{\sum }}\left(\overset{w_{ij},h_{ij}}{\underset{p,q=1}{\sum }}\frac{S_{pq}^{ij,k}}{w_{ij}h_{ij}}\right), \end{array}$$

where *𝒮*_*pq*_^*ij*,*k*^ = *𝒟*(*φ*_*i*,*j*_(*I*_*ℒ*_)_*pq*_ − *φ*_*i*,*j*_(*I*_*𝒮*_^*k*^)_*pq*_) and *φ*_*i*,*j*_ represents the feature map of the *j*-th feature channel of the *i*-th feature layer (after activation) [42], *N*_*i*_ is the number of feature channels in the *i*-th feature layer and *M* is the number of convolution layers, and *w*_*ij*_ and *h*_*ij*_ represent the size of the feature map in the VGG19 network. Here, *𝒟* is the error measure of the vgg/ResNet feature maps between the ground truth *I*_*ℒ*_ and prediction *I*_*𝒮*_^*k*^. The most widely used feature distances also contain the manhattan distance *𝒟*_manh_ and the cosine similarity *𝒟*_cosine_ difined by

(9) $$\begin{array}{c} D_{\text{manh}}\left(X,Y\right)=\sum {\left\|X-Y\right\|}_{1},\\ D_{\text{cosine}}\left(X,Y\right)=1-\frac{\left(X,Y\right)}{{\left\|X\right\|}_{2}{\left\|Y\right\|}_{2}}, \end{array}$$

where *X* and *Y* are feature maps.

The total proposed segmentation model is trained by jointly minimizing the total loss *ℒ*^*s*^ for the three parts as follows:

(10) $$\begin{array}{c} {\left(\left\{G_{1}^{s},\cdots ,G_{n}^{s}\right\},D^{s}\right)}^{*}=\arg\;\min\;\max_{\left(\left\{G_{1}^{s},\cdots ,G_{n}^{s}\right\},D^{s}\right)}\left\{L^{s}\left(\left\{G_{1}^{s},\cdots ,G_{n}^{s}\right\},D^{s}\right)≕\lambda_{l}L_{1}\left(G_{1}^{s},\cdots ,G_{n}^{s}\right)+L_{\text{gan}}\left(\left\{G_{1}^{s},\cdots ,G_{n}^{s}\right\},D^{s}\right)+\lambda_{\text{vgg}}L_{\text{vgg}}\left(I_{L},\left\{G_{1}^{s},\cdots ,G_{n}^{s}\right\}\right)\right\}, \end{array}$$

where the *λ*_*l*_ and *λ*_vgg_ are two given weight parameters.

## 4. Results and Discussion

The proposed CMMCSegNet framework is implemented using PyTorch. The experiments are conducted on a single GeForce RTX 2080Ti GPU with 11 GB RAM. To identify the model design, we performed several ablation experiments. They are described as follows.

### 4.1. Dataset and Experimental Setting

To demonstrate our CMMCSegNet framework, we use MS-CMRSeg 2019 datasets [1], which contain three different modalities: LGE with 45 patients but only 5 patients being labeled and bSSFP with 35 annotated patients and T2-weighted. The goal of CMR segmentation challenge is to achieve LGE image segmentation. Since there are fewer T2-weighted slices for each patient in the dataset (about 3-7 slices for each patient), we only use bSSFP modality and LGE modality in our experiments.

The cross-modality translation network is trained for 200 epochs, and the model that performs best on the validation set was selected for translation from LGE to bSSFP in the proposed CMMCSegNet framework. The dataset training the segmentation network contains two parts, most of them are from real annotated bSSFP images (slices from the 25 patients), and a small amount of fake bSSFP images are translated from the annotated LGE images (slices from about two patients) by the Cycle-GAN translation network.

We also train 200 epochs for the segmentation network. The both models are trained using Adam optimization with a minibatch size of 1, a decayed learning rate with an initial value 1.0*e* − 2, the size *n*_*D*_ = 70 of patch D in the discriminator based on Patch-GAN, and the weight hyperparameters *λ*_1_ = 10, *λ*_gan_ = 1, *λ*_*l*_ = 100, and *λ*_vgg_ = 1.

### 4.2. Performance of Cross-Modality Translation

We first use Cycle-GAN to achieve translation between LGE and bSSFP modalities; we also employ three evaluation metrics, including Structural Similarity (SSIM), Peak Signal To Noise Ratio (PSNR), and Mutual Information (MI), to evaluate the performance of Cycle-GAN translation network, which is tested on the whole LGE and bSSFP images. Many randomly chosen results from the translated (fake) LGE or bSSFP modalities are shown in Figure 3. In Table 1, our translation model also leads to a comparable synthesis quality between LGE and bSSFP modalities for the whole datasets, where *A*_*r*_, *A*_*f*_, *B*_*r*_, and *B*_*f*_ denote real LGE, fake LGE, real bSSFP, and fake bSSFP, respectively.

### 4.3. Comparisons for Different Choices of Adversarial Loss and Perceptual Loss

After the cross-modality translation, two fake bSSFP patients with annotated masks (obtained from the cross-modality translation of two LGE patients with the ground truth) and fully real labeled bSSFP patients (35 patients) are used to train our proposed segmentation network. Next, we did several different comparison experiments for segmentation evaluations of fake bSSFP without annotated data (obtained from the cross-modality translation).

Table 2 shows the dice score of cardiac LGE segmentation in using different adversarial losses (Vanilla GAN, LSGAN, and WGAN-GP) and different CMMCSegNet generator blocks (U-net and ResNet) and with/without perceptual loss (*ℒ*_manh_ or *ℒ*_cosine_). We can also see that the overall segmentation performance of the U-net generator is slightly better than that of the ResNet generator using 6 different losses in terms of the LV (left ventricle), MYO (myocardium), and RV (right ventricle). For the U-net generator, the model using LSGAN loss yields better diagnostic performance than those of both Vanilla GAN and WGAN-GP losses. Besides, the *ℒ*_manh_ perceptual loss or *ℒ*_cosine_ perceptual loss added for kernel feature comparisons can guarantee that the network learn relevant high feature levels and content features, which will improve the segmentation results for Vanilla GAN and LSGAN. However, the dice score of LV and RV segmentation slightly decreases when WGAN-GP with the *ℒ*_mannh_ perceptual loss is used, while in the ResNet generation network, the models with the perceptual loss (*ℒ*_mannh_ or *ℒ*_cosine_) achieve higher segmentation performance in all three terms and outperform those without the perceptual loss.

### 4.4. Comparisons of the Cascade Generators

High-level semantic features in each branch contain sufficient localization information of corresponding region. To make full use of the features, we propose the multicascade architecture to extract implicitly geometrical and textural information that guides the cardiac segmentation. In order to enhance the competitiveness of the proposed architecture, we evaluate the performances by running a pix2pix segmentation on the training dataset (real/fake bSSFP images with ground truths). Final results are achieved with an ensemble of 1-4 cascades using corresponding LSGAN's adversarial loss and perceptual loss. Comparisons with different number of cascades are shown in Table 3; we can see that the number of cascades is increased from one to four and the dice values of some terms dropped slightly for the model with/without perceptual loss. The reason for this may be that the increase in the number of cascades may cause a lot of edge information to be lost in the original fake bSSFP images. As we can see from Figure 1, when the first segmentation network *G*_1_^*s*^ obtains the segmentation result of the input fake bSSFP images, if original fake bSSFP image *I*_*𝒴*_ is not used as a conditional input in the later *G*_*k*+1_^*s*^, modifying the previous result *I*_*𝒮*_^*k*^, *G*_*k*+1_^*s*^ extracts fewer features comparing with the *G*_1_^*s*^. To optimize the computational costs, starting from the second generator, we reduce the number of upsampling/downsampling layers in the middle part of the U-net generators from (8, 8, 8) to (2, 4, 5) for generators (*G*_2_^*s*^, *G*_3_^*s*^, *G*_4_^*s*^), respectively. From Table 3, we observe that the proposed network with the simplified U-net versions can improve the segmentation results.  Figure 4 shows the original LGE images, the translated bSSFP images, the corresponding ground truths, and the prediction results with varying the numbers of cascades.

### 4.5. Comparisons of the Weights *ω*_*k*_^*ℒ*_*g*_^ and *ω*_*k*_^*ℒ*_1_^ of Multicascade Blocks

The performance of the multicascade architecture may be directly limited by the loss weight parameter of each cascade generator *G*_*k*_^*s*^. We compare the choice of the weights *ω*_*k*_^*ℒ*_*g*_^ and *ω*_*k*_^*ℒ*_1_^, and *I*_*S*_^*k*^ represents the output of the *k*-th generator *G*_*k*_^*s*^. From Table 4, the model with LSGAN adversarial loss and vgg perceptual loss is optimized solely using loss weights (*ω*_1_^*ℒ*_1_^, *ω*_2_^*ℒ*_1_^, *ω*_3_^*ℒ*_1_^) = (*ω*_1_^*ℒ*_*g*_^, *ω*_2_^*ℒ*_*g*_^, *ω*_3_^*ℒ*_*g*_^) = (1/3, 1/2, 1/6) and achieves the better results on the evaluation dice of *I*_*𝒮*_^2^. Due to the efficiency of the multicascade technique, the proposed segmentation network automatically improves image multilevel features that benefits the segmentation performance.  Figure 5 shows the results of different generators in a multicascade pix2pix network with different weights; *G*_2_^*s*^ can further modify the details of *I*_*𝒮*_^1^ making the output result closer to ground truth.

### 4.6. Comparison to Conventional Methods

Table 5 benchmarks the performance of the proposed framework against the direct and indirect LGE segmentation networks. First, we compare the performance of the four direct segmentation methods, including FCNs [4], U-net [5], U-net++ [44], and Attention U-net [45] networks by directly training a segmentation network from a small number of annotated LGE images. As reported in Table 5, although U-net performs better than others, it produces low dice value.  Figure 6(a) visualizes the segmentation results by direct methods. We also compare the performance of the five indirect segmentation methods, including FCNs, U-net, U-net++, and Attention U-net networks and the proposed CMMCSegNet by indirectly training networks from a small number of annotated fake bSSFP images and fully real bSSFP annotated images. As shown in Table 5, the proposed technique provides the highest dice score of LV and MYO and the fair value in RV. This means that our proposed CMMCSegNet outperforms the other techniques.  Figure 6(b) further illustrates a more detailed comparison between the proposed and other techniques; our proposed CMMCSegNet has obvious advantages that it is easier to learn the location information of the target area.

## 5. Conclusion

In this work, we proposed a CMMCSegNet framework based on multimodal cardiac MR images for indirect LGE segmentation. Firstly, we utilized Cycle-GAN to translate LGE modality into bSSFP modality and then segmented the translated (fake) bSSFP images to achieve indirect segmentation of LGE images. The advantage of this method is that only a small number of annotated LGE images can be required to achieve accurate segmentation of LGE by employing many annotated bSSFP images. This indirection also solved the problem of LGE images itself having a low contrast. Compared with the direct segmentation of LGE images, the indirect segmentation method has better segmentation performance.

For the multicascade pix2pix network, we regard the segmentation as a translation from image to ground truth; the purpose of multicascade architecture is to better improve the previous prediction through several generators. We also compared the use of different adversarial losses, the experimental results show LSGAN loss is better than the Vanilla GAN and WGAN-GP, and WGAN-GP loss is not significantly better than the Vanilla GAN loss. To improve the training effect of the model, the perceptual losses based on *ℒ*_manh_ and *ℒ*_cosine_ measures are also used to optimize the features of each feature layer. In addition, we investigated the influence of the weights of the generation loss of multicascade structures, where the optimal weight coefficient is set to (1/3, 1/2, 1/6) for 3 cascade generation networks.

We also demonstrated the effectiveness of the proposed CMMCSegNet by comparing with FCNs, U-net, U-net++, and Attention U-net. In the future, we will consider the end-to-end segmentation method to segment the multimodal cardiac MR, combining the translation and segmentation together.

## Figures and Tables

**Figure 1:** The proposed cross-modality multicascade SegNet flowchart of indirect segmentation for LGE modality. bSSFP images are important in distinguishing the cardiac structure from all enhanced areas. Accordingly, the two imaging modalities are treated differently in the proposed method. Cross-modality translation from LGE to bSSFP is chosen as Stage I of the proposed architecture having a greater impact on the LGE segmentation results. bSSFP is regarded as the assistant modality completing the LGE segmentation.

**Figure 2:** Different modalities of CMR imaging from the same patient (the two images are unpaired). LGE can enhance myocardial necrosis or scarring, which can evaluate effectively cardiac structure, cardiac function, myocardial perfusion, and myocardial activity, while bSSFP can highlight clearly the large blood vessels and coronary arteries because of more obvious contrast in the heart muscle and blood pool. To better adapt to cardiac structure segmentation, we will build a cross-modality translation network based on Cycle-GAN (Figure 1(b)).

**Figure 3:** Performance evaluations of Cycle-GAN cross-modality translation.

**Figure 4:** Qualitative comparisons of our CMMCSegNet for different number of cascade blocks on fake bSSFP translated from LGE modality. From left to right: LGE, bSSFP translated by Cycle-GAN, ground truth with zoom-in views, and prediction results with zoom-in views using 1-4 cascade blocks.

**Figure 5:** Comparisons of the loss weights of different cascade prediction *I*_*𝒮*_^*k*^ in proposed CMMCSegNet, where the LSGAN adversarial loss and vgg *ℒ*_manh_ perceptual loss are employed and the loss weight parameters (*ω*_1_^*ℒ*_1_^, *ω*_2_^*ℒ*_1_^, *ω*_3_^*ℒ*_1_^) = (*ω*_1_^*ℒ*_*g*_^, *ω*_2_^*ℒ*_*g*_^, *ω*_3_^*ℒ*_*g*_^) = (1/3, 1/2, 1/6) are manually given. (a) the LGE image and the corresponding ground truth; (b) from left to right: the predicted results {*I*_*𝒮*_^*k*^} under different loss weights (1/3, 1/3, 1/3), (1/6, 1/3, 1/2), (1/2, 1/3, 1/6), and (1/3, 1/2, 1/6), from top to bottom: *I*_*𝒮*_^1^, *I*_*𝒮*_^2^, *I*_*𝒮*_^3^.

**Figure 6:** Qualitative comparisons of our CMMCSegNet with the other four state-of-the-art CNN-based segmentation methods, where the LSGAN adversarial loss and vgg *ℒ*_manh_ perceptual loss are employed and the loss weight parameters (*ω*_1_^*ℒ*_1_^, *ω*_2_^*ℒ*_1_^, *ω*_3_^*ℒ*_1_^) = (*ω*_1_^*ℒ*_*g*_^, *ω*_2_^*ℒ*_*g*_^, *ω*_3_^*ℒ*_*g*_^) = (1/3, 1/2, 1/6) is manually given. (a) Direct segmentation, from left to right: LGE, ground truths with zoom-in views and prediction results with zoom-in views using FCNs, U-net, U-net++, and Attention U-net for segmentation on real LGE modality; (b) indirect segmentation, from left to right: LGE, fake bSSFP, ground truths with zoom-in views, and prediction results with zoom-in views using FCNs, U-net, U-net++, Attention U-net, and our CMMCSegNet for segmentation on fake bSSFP modality translated from LGE modality.

**Table 1:** Performance evaluations of Cycle-GAN cross-modality translation.

Translation	Evaluation	SSIM	PSNR	MI
*A*_*r*_⟶*B*_*f*_⟶*A*_*f*_	(*A*_*r*_, *A*_*f*_)	0.944	29.557	0.484
*B*_*r*_⟶*A*_*f*_⟶*B*_*f*_	(*B*_*r*_, *B*_*f*_)	0.962	28.911	0.493

**Table 2:** Indirect segmentation performance comparisons between CMMCSegNet models based on U-net and ResNet generator blocks using different training losses, where only one cascade generation block is used, “P-*ℒ*_cosine_” means to add cosine similarity perceptual loss into training loss, and “P-*ℒ*_manh_” means to add *ℒ*_manh_ perceptual loss into training loss.

Block	Loss	LV	MYO	RV
U-net	Vanilla GAN loss	0.8038 ± 0.2068	0.7463 ± 0.0534	0.8208 ± 0.0304
	Vanilla GAN loss + P‐*L*_cosine_	0.8575 ± 0.1153	0.7580 ± 0.0573	0.8459 ± 0.0306
	Vanilla GAN loss + P‐*L*_manh_	0.8815 ± 0.0833	0.7412 ± 0.0630	0.8600 ± 0.0279
	WGAN-GP loss	0.8420 ± 0.1068	0.7169 ± 0.0814	0.8448 ± 0.0584
	WGAN-GP loss + P‐*L*_cosine_	0.8162 ± 0.1106	0.7485 ± 0.0486	0.8563 ± 0.0349
	WGAN-GP loss + P‐*L*_manh_	0.8363 ± 0.1393	0.7436 ± 0.1204	0.8422 ± 0.0779
	LSGAN loss	0.8938 ± 0.0775	0.7542 ± 0.0601	0.8541 ± 0.0267
	LSGAN loss + P‐*L*_cosine_	0.9038 ± 0.0619	0.7513 ± 0.0739	0.8693 ± 0.0287
	LSGAN loss + P‐*L*_manh_	0.9018 ± 0.0674	0.7606 ± 0.0645	0.8631 ± 0.0362

ResNet	Vanilla GAN loss	0.8326 ± 0.1063	0.7486 ± 0.1019	0.8306 ± 0.0771
	Vanilla GAN loss + P‐*L*_cosine_	0.8762 ± 0.0812	0.7612 ± 0.0866	0.8524 ± 0.0246
	Vanilla GAN loss + P‐*L*_manh_	0.8787 ± 0.0977	0.7742 ± 0.0687	0.8568 ± 0.0210
	WGAN-GP loss	0.7665 ± 0.2210	0.7729 ± 0.0498	0.8357 ± 0.0299
	WGAN-GP loss + P‐*L*_cosine_	0.8158 ± 0.1355	0.7504 ± 0.0805	0.8710 ± 0.0236
	WGAN-GP loss + P‐*L*_manh_	0.8589 ± 0.1137	0.7804 ± 0.04781	0.8574 ± 0.0210
	LSGAN loss	0.8663 ± 0.1265	0.7406 ± 0.0982	0.8558 ± 0.0888
	LSGAN loss + P‐*L*_cosine_	0.8831 ± 0.0899	0.7533 ± 0.0775	0.8737 ± 0.0289
	LSGAN loss + P‐*L*_manh_	0.8814 ± 0.1109	0.7566 ± 0.1065	0.8534 ± 0.0966

**Table 3:** Performance comparisons for the number of cascade generators on the multicascade pix2pix segmentation network, where “P-*ℒ*_manh_” means to use *ℒ*_manh_ perceptual loss and “simple” means to use cascade generator with the simplified U-net version (where the number of upsampling/downsampling layers in the middle part of the U-net generators is reduced from (8, 8, 8) to (2, 4, 5) for generators (*G*_2_^*s*^, *G*_3_^*s*^, *G*_4_^*s*^), respectively).

Number of cascades	LV	MYO	RV
1	0.8938 ± 0.0775	0.7542 ± 0.0601	0.8541 ± 0.0267
+P-*L*_manh_	0.9018 ± 0.0674	0.7606 ± 0.0645	0.8631 ± 0.0362
2	0.8824 ± 0.0632	0.7608 ± 0.0647	0.8631 ± 0.0273
+P-*L*_manh_	0.8929 ± 0.0853	0.7690 ± 0.0662	0.8831 ± 0.0310
+P-*L*_manh_+simple	0.8966 ± 0.0808	0.7732 ± 0.0768	0.8841 ± 0.0295
3	0.8527 ± 0.0659	0.7202 ± 0.0911	0.8248 ± 0.0284
+P-*L*_manh_	0.8762 ± 0.0769	0.7901 ± 0.0538	0.8874 ± 0.0175
+P-*L*_manh_+simple	0.8931 ± 0.0557	0.7664 ± 0.0520	0.8739 ± 0.0299
4	0.8778 ± 0.0905	0.7899 ± 0.0545	0.8764 ± 0.0177
+P-*L*_manh_	0.8944 ± 0.0770	0.7561 ± 0.0735	0.8815 ± 0.0252
+P-*L*_manh_+simple	0.9019 ± 0.0634	0.7690 ± 0.0706	0.8911 ± 0.0233

**Table 4:** Performance comparisons of indirect segmentation prediction *I*_*𝒮*_^*i*^ with different generation loss weights and U-net block, where the LSGAN adversarial loss and vgg *ℒ*_manh_ perceptual loss are employed.

Loss weight	*I*_*𝒮*_^*i*^	LV	MYO	RV
(1/3, 1/3, 1/3)	*I*_S_^1^	0.8792 ± 0.0846	0.7855 ± 0.0601	0.8580 ± 0.0279
	*I*_S_^2^	0.8818 ± 0.0779	0.7960 ± 0.0574	0.8830 + 0.0215
	*I*_S_^3^	0.8762 ± 0.0769	0.7901 ± 0.0539	0.8874 ± 0.0176

(1/6, 1/3, 1/2)	*I*_S_^1^	0.8860 ± 0.0764	0.7569 ± 0.0849	0.8532 ± 0.0384
	*I*_S_^2^	0.8881 ± 0.0683	0.7668 ± 0.0791	0.8460 ± 0.0326
	*I*_S_^3^	0.8631 ± 0.0846	0.7661 ± 0.0895	0.8535 ± 0.0377

$\left(\frac{1}{2},\frac{1}{3},\frac{1}{6}\right)$	*I*_S_^1^	0.9001 ± 0.0714	0.7332 ± 0.0932	0.8481 ± 0.0369
	*I*_S_^2^	0.9039 ± 0.0661	0.7472 ± 0.0879	0.8669 ± 0.0344
	*I*_S_^3^	0.8973 ± 0.0686	0.7308 ± 0.0847	0.8640 ± 0.0346

$\left(\frac{1}{3},\frac{1}{2},\frac{1}{6}\right)$	*I*_S_^1^	0.9037 ± 0.0633	0.7410 ± 0.0799	0.8579 ± 0.0283
	*I*_S_^2^	0.9061 ± 0.0593	0.7459 ± 0.0853	0.8733 ± 0.0273
	*I*_S_^3^	0.8726 ± 0.0585	0.7204 ± 0.0888	0.8513 ± 0.0214

**Table 5:** Performance comparisons between direct and indirect segmentation of LGE modality using different techniques, where the LSGAN adversarial loss and vgg *ℒ*_manh_ perceptual loss are employed and the loss weight parameters (*ω*_1_^*ℒ*_1_^, *ω*_2_^*ℒ*_1_^, *ω*_3_^*ℒ*_1_^) = (*ω*_1_^*ℒ*_*g*_^, *ω*_2_^*ℒ*_*g*_^, *ω*_3_^*ℒ*_*g*_^) = (1/3, 1/2, 1/6) are manually given.

Strategy	Network	LV	MYO	RV
Direct	FCNs [4]	0.4223 ± 0.2124	0.4696 ± 0.2174	0.6020 ± 0.2908
	U-net [5]	0.5746 ± 0.3062	0.4475 ± 0.2576	0.6876 ± 0.2291
	U-net++ [44]	0.5534 ± 0.3467	0.4294 ± 0.3541	0.6208 ± 0.3098
	Attention U-net [45]	0.6022 ± 0.1596	0.4544 ± 0.2376	0.6698 ± 0.2328

Indirect	FCNs [4]	0.7595 ± 0.1321	0.6113 ± 0.1689	0.8731 ± 0.0677
	U-net [5]	0.8505 ± 0.0991	0.7708 ± 0.0765	0.9151 ± 0.0441
	U-net++ [44]	0.8459 ± 0.1060	0.7470 ± 0.1030	0.9163 ± 0.0409
	Attention U-net [45]	0.8438 ± 0.1060	0.7593 ± 0.0953	0.9133 ± 0.0355
	CMMCSegNet	0.8762 ± 0.0769	0.7901 ± 0.05386	0.8874 ± 0.0176

## Data Availability

Dataset is obtained from Multisequence Cardiac MR Segmentation Challenge (MS-CMRSeg 2019; https://zmiclab.github.io/mscmrseg19/). This challenge is aimed at creating an open and fair competition for various research groups to test and validate their methods, particularly for the multisequence ventricle and myocardium segmentation. Also refer to publication [1].
